The article "Dendrobium Mixture Ameliorates Diabetic Nephropathy in db/db Mice by Regulating the TGF-β1/Smads Signaling Pathway" was published in 2021. Journal: Evid Based Complement Alternat Med.

# *Dendrobium* Mixture Ameliorates Diabetic Nephropathy in db/db Mice by Regulating the TGF-*β*1/Smads Signaling Pathway

**DOI:** 10.1155/2021/9931983

**Published:** 2021-09-30

**Authors:** Yong Chen, Xiaohui Lin, Yanfang Zheng, Wenzhen Yu, Fan Lin, Jieping Zhang

**Affiliations:** ^1^College of Integrated Traditional Chinese and Western Medicine, Fujian University of Traditional Chinese Medicine, Fuzhou 350122, China; ^2^College of Pharmacy, Fujian University of Traditional Chinese Medicine, Fuzhou 350122, China

## Abstract

*Dendrobium* mixture (DMix) is an effective treatment for diabetic nephropathy (DN), but the molecular mechanism underlying its action remains unclear. In this study, we investigated whether DMix regulates the transforming growth factor-*β*1 (TGF-*β*1)/Smads signal transduction pathway. Twenty-four db/db mice were randomly divided into three groups: the model, DMix, and gliquidone groups, while eight db/m mice were selected as the normal control group. The drug was administered by continuous gavage for 8 weeks. Body weight (BW), kidney weight (KW), kidney index, fasting blood glucose (FBG), blood lipid, 24-hour urinary albumin excretion rate, blood urea nitrogen, and serum creatinine levels were measured. Pathological changes in the renal tissue were observed under a light microscope. Real-time quantitative PCR and immunohistochemical staining were used to detect the mRNA and protein expression levels of TGF-*β*1 and alpha-smooth muscle actin (*α*-SMA), respectively, in renal tissues. TGF-*β*1, Smad2, p-Smad2, Smad3, p-Smad3, and *α*-SMA expression levels were measured using western blotting. The results showed that DMix significantly reduced the FBG level, BW, KW, and blood lipid level and improved renal function in db/db mice. Histopathology showed that DMix alleviated glomerular mesangial cell proliferation and renal interstitial fibrosis in db/db mice. Additionally, DMix reduced the protein and mRNA expression levels of TGF-*β*1 and *α*-SMA and inhibited Smad2 and Smad3 phosphorylation. We conclude that DMix may inhibit renal fibrosis and delay the progression of DN by regulating the TGF-*β*1/Smads signaling pathway.

## 1. Introduction

Diabetic nephropathy (DN) is a common chronic microvascular complication of diabetes and the most important cause of death in patients with diabetes [1, 2]. DN is characterized by the thickening of the glomerular basement membrane, proliferation of mesangial cells, and accumulation of extracellular matrix, leading to glomerulosclerosis and interstitial fibrosis [3, 4]. Transforming growth factor-*β*1 (TGF-*β*1) is a key cytokine-promoting fibrosis, and the Smad protein is the intracellular kinase substrate of the TGF-*β*1 receptor, mediating the TGF-*β*1 signaling pathway. Activation of the TGF-*β*1/Smads signal transduction pathway is an important mechanism for the development of renal fibrosis [5–7]. *Dendrobium* mixture (DMix) is a preparation used at the Second Affiliated Hospital of Fujian Traditional Chinese Medical University (batch number: Min Q/YZ-2012-315; patent number: ZL201110408411.0) that was developed by Professor Shi Hong for the long-term clinical treatment of diabetes and its complications. It is composed of *Dendrobium*, *Astragalus*, *Salvia miltiorrhiza*, *Rhizoma anemarrhenae*, and other herbs. It has the effects of lowering glucose and lipid levels and improving insulin resistance following clinical application [8–10], but the potential molecular mechanism remains unclear. In this study, the effect of DMix on the TGF-*β*1/Smads signaling pathway in the renal tissue of db/db mice with DN was observed, and the mechanism by which it improves DN was discussed to provide an experimental basis for the use of DMix in clinical practice.

## 2. Materials and Methods

### 2.1. Drug

DMix decoction, consisting of 15 g *Dendrobium*, 20 g *Astragalus,* 8 g *Schisandra*, 15 g *Radix puerariae*, 20 g *Salvia miltiorrhiza*, 18 g *Rehmanniae*, and 12 g *Rhizoma anemarrhenae*, was purchased from Guoyitang Clinic, Fujian University of Traditional Chinese Medicine (FJTCM). Gliquidone tablets (batch no. 1140573) were purchased from Beijing Wanhui Shuanghe Pharmaceutical Co., Ltd, Beijing, China.

### 2.2. Animals

*db/db* Mice (male, 11 weeks old, weight 42–46 g) and *db/m* mice (male, 11 weeks old, weight 21–24 g) were provided by the Department of Experimental Animal Science, Beijing University Medical Science Department (license number: SCXK (Jing) 2011-0012) and kept in a specific-pathogen-free environment at the Experimental Animal Center, FJTCM, with free access to standard diet and water. All animal experiments were conducted in accordance with internationally recognized animal welfare guidelines and approved by the medical ethics committee of FJTCM (approval no. 2019-034).

### 2.3. Experimental Design

After 1 week of adaptive feeding, according to the fasting blood glucose (FBG) level and body weight (BW), db/db mice were randomly divided into three groups (*n* = 8): the model group, the DMix group, and the gliquidone group (positive control). In addition, eight db/m mice of the same age with normal performance were selected as the normal control group. All animals were administered the treatments through intragastric administration at the clinical equivalent dose for a 60 kg adult human. Mice in the normal control and model groups were administered 20 mL/(kg·d) normal saline, the positive control group received 5 mg/(kg·d) gliquidone, and the DMix treatment group received 12 g/(kg·d) DMix, once a day for 8 weeks.

### 2.4. Measurement of FBG Level, BW, Kidney Weight (KW), Kidney Index (KI), Blood Lipid Level, and Renal Function

The FBG level of the mice was measured with a blood glucose meter and a test paper once every 2 weeks during treatment, using blood collected at the tail tip. After 8 weeks of administration, the weight of the mice was determined, and the mice were placed into a metabolic cage. Urine was collected for 24 hours, and the urinary albumin excretion rate (UAER) was determined using a urine protein quantitative kit (Nanjing Jiancheng Bioengineering Institute, Nanjing, China). After treatment, all mice were anesthetized via an intraperitoneal injection of 2% sodium pentobarbital (0.01 mL/g). Orbital blood was collected to separate the serum for the detection of blood urea nitrogen (BUN), serum creatinine (Scr), total cholesterol (TC), and triglyceride (TG) levels. All biochemical analysis kits were purchased from Nanjing Jiancheng Bioengineering Institute (Nanjing, China). After the mice were sacrificed, both kidneys were removed, washed with normal saline, and weighed.

### 2.5. Renal Histology

A part of the kidney tissue was fixed in 4% paraformaldehyde solution, embedded in paraffin, cut into 4 *μ*m-thick sections, and then stained with hematoxylin-eosin (HE), periodic acid-Schiff (PAS), and Masson. The stained kidney sections were examined under a light microscope at a magnification of ×400. The mean glomerular area, the ratio of mesangial matrix area to total glomerular area in PAS-stained sections, and the ratio of collagen accumulation area to total glomerular area in Masson trichromatic stained sections were measured using ImagePro Plus 6.0 quantitative software. In each section, ten glomeruli were randomly selected, the positive signals in the selected glomeruli were highlighted and measured, and the positive areas were quantified as a percentage of the entire glomerulus.

#### 2.5.1. HE Staining

The dried kidney tissue sections were dewaxed using xylene, graded alcohol, and distilled water, then stained with hematoxylin for 10 min, differentiated with 1% hydrochloric acid alcohol for 5 s, and then put into eosin for 3 min. Then, dehydration and transparent sealing were performed before observation under a light microscope.

#### 2.5.2. PAS Staining

The dried kidney tissue sections were dewaxed using xylene, graded alcohol, and distilled water followed by iodic acid oxidation solution for 5 min and Schiff reagent for 15 min. After hematoxylin staining for 1 min, 1% hydrochloric acid alcohol differentiation for 3 s, dehydration, and transparent sealing were performed for microscopic examination.

#### 2.5.3. Masson Staining

Dried kidney tissue sections were dewaxed using xylene, gradient alcohol, and distilled water and then fixed for 1 h in Bouin fixative solution. Masson composite dyeing solution was soaked for 10 min, and the 1% phosphomolybdate was separated for 10 min. The collagen fiber showed a reddish color and was soaked in 2% aniline blue solution for 5 min. Then, dehydration and transparent sealing were performed before observation under a light microscope.

### 2.6. Real-Time Quantitative PCR (RT-qPCR)

Total RNA was extracted from mice kidney tissue with RNAiso Plus reagent (Takara, Tokyo, Japan), and the concentration was determined. Then, cDNA was synthesized by reverse transcription using a reverse transcription kit (Takara, Tokyo, Japan). The PCR reaction was performed using a PCR kit (Takara, Tokyo, Japan) under the following reaction conditions: initial denaturation at 95°C for 30 s, followed by 40 cycles of denaturation at 95°C for 5 s, annealing at 55°C for 30 s, and extension at 72°C for 1 min. SDS 2.4 software was used to analyze the CT values of the samples detected during the PCR process, using *β*-actin as the internal reference and adopting the ΔΔCt method for relative quantitative analysis, with 2^−△△Ct^ as a quantity relative expression of the target RNA. PCR primers (Table 1) were designed and provided by Fuzhou Shangya Biotechnology Co., Ltd (Fuzhou, China).

### 2.7. Immunohistochemistry

The kidney tissue was fixed in 4% paraformaldehyde solution, embedded in paraffin, cut into 4 *μ*m-thick slices, baked for 2 h, dewaxed using xylene twice, hydrated with gradient alcohol, placed into boiled sodium citrate solution for antigen repair, and cooled naturally to room temperature (18–30°C). The sections were rinsed with phosphate-buffered saline (PBS) thrice, co-incubated with an endogenous peroxidase blocker at room temperature for 10 min, rinsed with PBS thrice, and co-incubated with nonimmunized animal serum at room temperature for 10 min. After removing the serum, primary antibodies were added dropwise as follows: rabbit anti-TGF-*β*1 and anti-*α*-SMA polyclonal antibodies (1 : 100 dilution each; Abcam, Cambridge, UK), incubated at 4°C overnight and rinsed with PBS thrice; biotin-labeled sheep anti-rabbit IgG (ready to use, Fuzhou Maixin Biotech Co., Ltd, Fuzhou, China), incubated at room temperature for 10 min and rinsed with PBS thrice; and streptavidin-peroxidase (Fuzhou Maixin Biotech Co., Ltd, Fuzhou, China), incubated at room temperature for 10 min and rinsed with PBS thrice. DAB (Wuhan Boster Biological Technology Co., Ltd, Wuhan, China) was then added for color development, rinsed with distilled water, hematoxylin-dyed, and tap water-rinsed for blueness. The tissues were dehydrated using an alcohol gradient and subsequently dried, after which they were made transparent with xylene and sealed with neutral gum. Tissue sections were then assessed for positive staining (brown in color) under an optical microscope. The Image-Pro Plus 6.0 image analysis software was used for semiquantitative analysis; ten nonrepeated high-magnification (×400) visual fields containing glomeruli were randomly selected from each section to calculate the cumulative optical density (IOD) of the positive staining and the area of the measured section (area); the average values were then used for analysis, and the relative protein expression was represented by mean density (IOD/area).

### 2.8. Western Blot Assays

Kidney tissues stored in liquid nitrogen mixed with appropriate protein lysate were fully ground to produce tissue homogenates. After centrifugation (4°C, 12,000 rpm, 15 min), the total protein was extracted from the supernatant and the protein concentration was determined using the bicinchoninic acid assay. Then, 30 *μ*g of each sample was used for 10% SDS-PAGE gel electrophoresis, transferred to a polyvinylidene fluoride membrane, and sealed with 5% skim milk at room temperature for 1 h. Primary antibodies (TGF-*β*1, Smad2, p-Smad2, Smad3, p-Smad3, and *α*-SMA) were added and incubated with the membrane overnight at 4°C. After rinsing with tris-buffered saline, 0.1% Tween 20 (TBST), the membrane was incubated with the secondary antibody at room temperature for 1 h. After TBST rinsing, the membrane was stained using enhanced chemiluminescence and viewed using a gel imaging system. The corresponding antibody dilutions were as follows: *β*-actin (1 : 1000 dilution; Abcam, Cambridge, UK), TGF-*β*1 (1 : 500 dilution; Abcam, Cambridge, UK), Smad2 (1 : 1000 dilution; Abcam, Cambridge, UK), p-Smad2 (1 : 300 dilution; Abcam, Cambridge, UK), Smad3 (1 : 5000 dilution; Abcam, Cambridge, UK), p-Smad3 (1 : 2000 dilution; Abcam, Cambridge, UK), *α*-SMA (1 : 500 dilution; Abcam, Cambridge, UK), goat-anti-mouse IgG secondary antibody (1 : 2000 dilution; Beyotime, Shanghai, China), and goat-anti-rabbit IgG secondary antibody (1 : 1000 dilution; Beyotime, Shanghai, China). The gray value of the strip was measured using the Image Lab analysis software, and the results are expressed in terms of the relative expression of the target protein, using *β*-actin as the internal reference.

### 2.9. Statistical Analyses

SPSS 22.0 statistical software was used to analyze the data, which are expressed as mean ± standard deviation (SD). Differences among multiple sample groups were analyzed using one-way ANOVA. The Bonferroni method was used for pairwise comparison between groups when the variances were homogeneous, and Tamhane's T2 comparison was used when the variances were heterogeneous. *P* < 0.05 was considered statistically significant.

## 3. Results

### 3.1. Comparison of General Signs

Mice in the normal group were in a good mental state, responsive, with shiny hair, and in a good feeding condition. db/db mice were listless and unresponsive, with increased diet and urine volumes; the above symptoms of mice in each treatment group were improved to different degrees compared with the model group.

### 3.2. DMix Reduced Fasting Blood Glucose Levels of db/db Mice

The FBG level in *db/db* mice was approximately 3× higher than that in the normal group (*P* < 0.01). The FBG level in the DMix group gradually decreased with increasing treatment duration (Figure 1). After the 4th week, there was a significant reduction in the FBG level in the DMix group compared with the model group (week 4, *P* < 0.05; weeks 6 and 8, *P* < 0.01), and no statistically significant difference was observed between the DMix and positive control groups (*P* > 0.05), indicating that DMix could reduce blood glucose in db/db mice.

### 3.3. Comparison of BW, KW, and KI in Each Group

The BW, KW, and KI of *db/db* mice were significantly higher than those of the normal group (*P* < 0.05, *P* < 0.01). After 8 weeks of DMix treatment, the BW, KW, and KI of the mice were all lower than those of the model group to different degrees (KI, *P* < 0.05; BW and KI, *P* < 0.01) (Figure 2(a)–2(c)). Additionally, there was no significant difference between the DMix and gliquidone groups (*P* > 0.05).

### 3.4. Effects of DMix on TC and TG Levels in *db/db* Mice

The serum TC and TG levels of mice in the model group were significantly higher than those in the normal group (*P* < 0.01). TC and TG levels in both the DMix and gliquidone groups were significantly lower than those in the model group (TG, *P* < 0.05; TC, *P* < 0.01) (Figure 3(a) and 3(b)). There was no significant difference between the DMix and gliquidone groups (*P* > 0.05). These results indicate that DMix could regulate lipid metabolism.

### 3.5. DMix Improved Renal Function of db/db Mice

Renal function indices of mice in each group were measured, including Scr, BUN, and UAER. These indices were significantly higher in the model group than in the normal group (*P* < 0.01), indicating that the DN mouse model was successfully established and renal insufficiency was achieved in the DN mice. The Scr, BUN, and UAER levels of mice in the DMix group were significantly lower than those in the model group (*P* < 0.05), but there was no significant difference between the DMix and gliquidone groups (*P* > 0.05) (Figure 4(a)–4(c)). These results indicate that DMix had a protective effect on the kidney of db/db mice.

### 3.6. Effect of DMix on Renal Pathological Morphology of db/db Mice

HE (Figure 5(a)) and PAS (Figure 5(b)) staining showed clear renal tissue structure, normal glomerular size, morphology, and interstitial space, no increase in mesangial matrix size, unobstructed renal tubular lumen, intact epithelial cells, and no glycogen deposition. db/db mice had glomerular hypertrophy, a larger mesangial matrix, a wider mesangial region, partial capillary lumen stenosis, vacuolar degeneration of renal tubular epithelial cells, more renal mesenchymal cells, and large amounts of red-stained glycogen deposition. Both the DMix and gliquidone groups improved compared with the model group, with thinner glomerular basement membranes, significantly less mesangial cell proliferation, smaller extracellular matrix, and less glycogen deposition than in the model group. Additionally, in the DMix and gliquidone groups, the tubular structure of the kidney was nearly restored to normal. Masson staining (Figure 5(c)) showed collagen fiber accumulation in the glomerular and tubulointerstitial lesions of mice in the model group, and collagen fiber deposition improved significantly after DMix treatment. According to the quantitative analysis results, the glomerular area, percentage of mesangial matrix, and percentage of collagen accumulation area in the model group were significantly increased compared with the control group (*P* < 0.01). After 8 weeks of treatment, the glomerular area, the percentage of mesangial matrix, and the percentage of collagen accumulation decreased significantly compared with the model group (*P* < 0.05, *P* < 0.01). No significant difference was observed between the DMix and gliquidone groups (*P* > 0.05) (Figure 5(d)–5(f)).

### 3.7. DMix Inhibited the mRNA and Protein Expression Levels of TGF-*β*1 and *α*-SMA in the Renal Tissues of db/db Mice

TGF-*β*1 has been identified as a potential target for DN therapy, while the levels of *α*-SMA, a marker participating in the renal tubular epithelial-mesenchymal transition (EMT) process, are thought to reflect the degree of renal fibrosis [11, 12]. To evaluate the therapeutic effect of DMix, the mRNA expression levels of TGF-*β*1 and *α*-SMA were measured in renal tissues using RT-qPCR. Results show that the expressions of TGF-*β*1 and *α*-SMA in renal tissues of mice in the model group were significantly higher than those in the normal group (*P* < 0.01). Moreover, the expressions of TGF-*β*1 and *α*-SMA in the DMix and gliquidone groups were lower than those in the model group (*α*-SMA, *P* < 0.05; TGF-*β*1, *P* < 0.01); however, they remained higher than those in the normal group (Figure 6(a)). Moreover, no significant differences were observed between the DMix and gliquidone groups (*P* > 0.05), indicating that DMix inhibited the mRNA expression of TGF-*β*1 and *α*-SMA in renal tissues of *db/db* mice.

To further demonstrate the therapeutic effect of DMix, immunohistochemical staining was performed to detect the abundance of TGF-*β*1 and *α*-SMA proteins in the renal tissues of mice. The results were consistent with those of RT-qPCR. TGF-*β*1 and *α*-SMA were weakly expressed in the kidneys of mice in the normal group and strongly expressed in the model group (TGF-*β*1, *P* < 0.05; *α*-SMA, *P* < 0.01); brown positive staining was primarily detected in the epithelial cells of the glomeruli and renal tubules. The abundance of TGF-*β*1 and *α*-SMA was significantly lower in both treatment groups compared with the model group (*P* < 0.05); however, it remained higher than that in the normal group (Figures 6(b)–6(d)). Meanwhile, no significant difference was observed between the DMix and gliquidone groups (*P* > 0.05), indicating that DMix reduced the abundance of TGF-*β*1 and *α*-SMA proteins in the renal tissues of db/db mice.

### 3.8. DMix Inhibited the TGF-*β*1/Smads Signaling Pathway in the Renal Tissues of db/db Mice

The activation of the Smad pathway and its subsequent nuclear transposition is a key step in TGF-*β*1-mediated renal fibrosis in DN [13]. The phosphorylation of Smad2 and Smad3 is also an important signal transduction process in the TGF-*β*1/Smads signaling pathway, and their expression indicates TGF-*β*1/Smads signaling pathway activation [14]. The expression of TGF-*β*1, Smad2, p-Smad2, Smad3, p-Smad3, and *α*-SMA in mouse renal tissues was measured via western blotting. The protein expression of TGF-*β*1, p-Smad2, p-Smad3, and *α*-SMA in the model group was significantly higher than that in the normal group (*P* < 0.01), indicating that the TGF-*β*1/Smads signaling pathway was activated in db/db mouse renal tissue. After 8 weeks of treatment with DMix, the expression of TGF-*β*1, p-Smad2, p-Smad3, and *α*-SMA proteins was significantly lower than that in the model group (TGF-*β*1:*β*-actin, p-Smad2:Smad2, and *α*-SMA:*β*-actin, *P* < 0.05; p-Smad3:Smad3, *P* < 0.01), but there was no significant change in the expression of the Smad2 and Smad3 proteins (Figure 7(a)–7(d)). There was no significant difference between the DMix and gliquidone groups (*P* > 0.05). Western blots show that DMix inhibited the TGF-*β*1/Smads signaling pathway in the renal tissues of db/db mice.

## 4. Discussion

Currently, DN poses a great threat to human health, and traditional Chinese medicine has achieved good efficacy in the treatment of DN. In preliminary experimental studies and clinical practice, DMix has been shown to have a good therapeutic effect on diabetes mellitus and its complications [8–10, 15–17]. In this study, we observed that DMix can treat DN by inhibiting renal fibrosis and improving renal function. DMix reduced the expression of TGF-*β*1 and *α*-SMA and inhibited the phosphorylation of Smad2 and Smad3, thereby slowing DN progression.

DN is caused by a variety of factors, including hyperglycemia, hypertension, and hyperlipidemia [18–20]. The db/db mouse is a widely used animal model for the study of DN, and the pathogenesis is caused by a deficiency of the leptin receptor gene [21, 22]. The results of this experiment showed that db/db mice had a significantly greater body weight than db/m mice. Additionally, blood glucose, Scr and BUN levels, and KI were significantly higher in db/db mice than in the normal group. Furthermore, the db/db mice exhibited proteinuria, dyslipidemia, glomerular hypertrophy, and fibrosis, confirming that the DN model was successful. After treatment with DMix, these parameters were significantly attenuated (Figures 1–4), which was consistent with previous studies and our clinical observation [9–11]. Additionally, HE, PAS, and Masson staining showed that the degree of renal pathological injury and fibrous hyperplasia improved significantly in the model group with the administration of DMix (Figure 5). DN is characterized by proteinuria and glomerular sclerosis [23, 24], and our results indicate that DMix not only reduces urinary protein levels but also reduces renal fibrosis, suggesting that DMix effectively prevents the development of DN.

The pathogenesis of DN is complex and has not been fully elucidated. Renal interstitial fibrosis is an important mechanism of renal deterioration in the pathogenesis of DN. Therefore, the key to delay the development of DN is to inhibit renal interstitial fibrosis [25, 26]. TGF-*β*1/Smads is the core pathway of renal fibrosis and one of the important factors in the development of DN [27, 28]. TGF-*β*1 is considered an important factor contributing to renal mesenchymal fibrosis, and previous studies have confirmed that TGF-*β*1 is overexpressed in DN [29, 30]. Smad2 and Smad3 act downstream of TGF-*β*1, which promotes Smad2 and Smad3 phosphorylation when activated. Both proteins, which have a high homology, are subsequently transferred to the nucleus and regulate the expression of fibrosis-related target genes, such as *α*-SMA, to accelerate the progression of fibrosis [31–33]. The expression of p-Smad2 and p-Smad3 proteins is a marker of TGF-*β*1/Smads signaling pathway activation [34, 35]. Studies have shown that p-Smad2 and p-Smad3 expression levels increase significantly in patients with chronic kidney disease and animal models of renal fibrosis, thereby activating the TGF-*β*1/Smads signaling pathway and simultaneously increasing the expression of *α*-SMA protein, a marker of mesenchymal cells, the expression level of which reflects the degree of renal fibrosis [36–38]. The inhibition of the TGF-*β*1/Smads signaling pathway can effectively reduce DN renal fibrosis and improve renal function [39, 40]. In this study, immunohistochemical (Figure 6(b)–6(d)) and western blot (Figure 7) analyses showed that the expression levels of TGF-*β*1, p-Smad2, p-Smad3, and *α*-SMA proteins decreased significantly in the DMix group. The mRNA expression of TGF-*β*1 and *α*-SMA (Figure 6(a)) was consistent with the protein expression of TGF-*β*1 and *α*-SMA. These results suggest that DMix may inhibit renal fibrosis owing to DN by negatively regulating the TGF-*β*1/Smads pathway.

The treatment of diabetic complications focuses on early prevention. There are many types of drugs for the clinical treatment of DN. Effectively reducing blood glucose and avoiding nephrotoxicity are important selection basis. Gliquidone is recommended for oral treatment in the early stage of DN and was, therefore, used as a positive control in the current study because it can promote insulin secretion by binding to specific receptors on pancreatic cell membrane and exerts a certain renal protective effect [41]. In our study, we observed that both DMix and gliquidone reduced the blood glucose levels of db/db mice, inhibited the TGF-*β*1/Smads signaling pathway, and improved the renal function and pathological structure in the model animals. Previous studies have shown that high-glucose environment increases the expression of TGF-*β*1 in the kidney and activates the TGF-*β*1/Smads signaling pathway during the development of diabetes, which is closely related to the evolution of diabetic nephropathy [42, 43]. Therefore, we speculate that DMix can reduce the blood glucose level and inhibit the TGF-*β*1/Smads pathway, which may represent an important mechanism employed by DMix in the prevention and treatment of DN.

Although the results confirmed our hypothesis, our study may have had some limitations. For example, although DMix had an effect on DN renal fibrosis, more and larger studies and clinical trials are needed for further verification. Additionally, owing to time and financial constraints, we could not carry out cellular experiments to investigate the effect of DMix on DN, and the specific mechanism still needs to be studied.

## 5. Conclusion

Our results show that DMix exerts a protective effect on the kidneys of DN mice, which may be to inhibit renal EMT and fibrosis by regulating the TGF-*β*1/Smads pathway, thereby delaying the progression of DN. Therefore, DMix may be a promising drug for DN treatment.

## Figures and Tables

**Figure 1:** Eight weeks post-DMix treatment, fasting blood glucose of the normal (Control), model (Model), DMix (DMix), and gliquidone (Gliquidone) groups were tested. Data are presented as mean ± SD of eight animals for each group (*n* = 8). ^*∗∗*^*P* < 0.01 versus Control; ^#^*P* < 0.05 versus Model; ^##^*P* < 0.01 versus Model.

**Figure 2:** Changes in body weight (a), kidney weight (b), and kidney index (c) after DMix treatment. Data are presented as mean ± SD from eight animals for each group (*n* = 8). ^*∗∗*^*P* < 0.01 versus Control; ^#^*P* < 0.05 versus Model; ^##^*P* < 0.01 versus Model.

**Figure 3:** Values are expressed as mean ± SD of eight samples from each group (*n* = 8). ^*∗∗*^*P* < 0.01 versus Control; ^#^*P* < 0.05 versus Model; ^##^*P* < 0.01 versus Model.

**Figure 4:** Values are expressed as mean ± SD of eight samples from each group (*n* = 8). ^*∗∗*^*P* < 0.01 versus Control; ^#^*P* < 0.05 versus Model; ^##^*P* < 0.01 versus Model.

**Figure 5:** Photomicrographs of hematoxylin and eosin (a), periodic Acid-Schiff (b), and Masson (c) staining of mice kidneys from each group as observed under a light microscope (×400). Changes in glomerular area (d), the percentage of mesangial matrix (e), and the percentage of collagen area (f). Kidney tissue in the model group shows markedly severe destruction in the glomerular and tubulointerstitial lesions, including glomerular hypertrophy, increased mesangial matrix, interstitial cell infiltration, and collagen fiber deposition. After treatment, the overall morphology of the glomerular and tubulointerstitial lesions significantly improved. ^*∗∗*^*P* < 0.01 versus Control; ^#^*P* < 0.05 versus Model; ^##^*P* < 0.01 versus Model.

**Figure 6:** DMix suppressed TGF-*β*1 and *α*-SMA mRNA expression and protein levels in murine kidneys. mRNA levels of TGF-*β*1 and *α*-SMA (a), determined using RT-qPCR with *β*-actin as the internal standard for each sample. Immunohistochemical staining for TGF-*β*1 (b) and *α*-SMA (c) (×400); mean density of TGF-*β*1 and *α*-SMA (d). Relative TGF-*β*1 and *α*-SMA mRNA and protein expression levels after analysis. ^*∗*^*P* < 0.05 versus Control; ^*∗∗*^*P* < 0.01 versus Control; ^#^*P* < 0.05 versus Model; ^##^*P* < 0.01 versus Model.

**Figure 7:** DMix inhibits the renal TGF-*β*1/Smads signaling pathway in db/db mice, as shown using western blotting. *β*-Actin, Smad2, and Smad3 were used as internal standards. The relative expression were the ratios of TGF-*β*1:*β*-actin (a), p-Smad2:Smad2 (b), p-Smad3:Smad3 (c), and *α*-SMA:*β*-actin (d), determined via densitometric analysis. ^*∗∗*^*P* < 0.01 versus Control; ^#^*P* < 0.05 versus Model; ^##^*P* < 0.01 versus Model.

**Table 1:** RT-qPCR primers.

Gene name	Primer sequence	Product length (bp)
TGF-*β*1	Forward: 5′-CCAGATCCTGTCCAAACTAAGG-3′	169
	Reverse: 5′-CTCTTTAGCATAGTAGTCCGCT-3′	

*α*-SMA	Forward: 5′-GGACGTACAACTGGTATTGTGC-3′	179
	Reverse: 5′-TCGGCAGTAGTCACGAAGGA-3′	

*β*-actin	Forward: 5′-GTGACGTTGACATCCGTAAAGA-3′	245
	Reverse: 5′-GCCGGACTCATCGTACTCC-3′	

## Data Availability

The data used to support the findings of this study are included within the article.
